The article "A Simple RFLP-Based Method for HFE Gene Multiplex Amplification and Determination of Hereditary Hemochromatosis-Causing Mutation C282Y and H63D Variant with Highly Sensitive Determination of Contamination" was published in 2020. Journal: Biomed Res Int.

# A Simple RFLP-Based Method for *HFE* Gene Multiplex Amplification and Determination of Hereditary Hemochromatosis-Causing Mutation C282Y and H63D Variant with Highly Sensitive Determination of Contamination

**DOI:** 10.1155/2020/9396318

**Published:** 2020-12-28

**Authors:** Ludmilla OGOUMA-AWORET, Jean-Pierre RABES, Philippe de MAZANCOURT

**Affiliations:** ^1^Laboratory of Biochemistry and Molecular Genetics, Hospital Ambroise Paré-GHU APHP, Université Paris-Saclay, Boulogne-Billancourt, France; ^2^UMR1179, INSERM/UVSQ, France

## Abstract

Hereditary hemochromatosis is an autosomal recessive disorder with incomplete penetrance that results from excess iron absorption and can lead to chronic liver disease, fibrosis, cirrhosis, and hepatocellular carcinoma. The most common form of hereditary hemochromatosis in Western Europe is due to a homozygous mutation (p.(Cys282Tyr) or C282Y), in the *HFE* gene which encodes hereditary haemochromatosis protein. In the general European population, the frequency of the homozygous genotype is 0.4%, and this mutation explains up to 95% of hereditary hemochromatosis in France. We report here an improved PCR and restriction endonuclease assay based on multiplex amplification of *HFE* exon 4 (for C282Y detection), *HFE* exon 2 (for H63D detection), *FZD1* gene (for digestion controls), and two Short Tandem Repeats (SE33 and FGA) for identity monitoring and contamination tracking. Fluorescent primers allow capillary electrophoresis, accurate allele tagging, and sensitive contamination detection.

## 1. Introduction

Patients with hemochromatosis are characterized by progressive accumulation of iron in parenchymal tissues, primarily the liver. In *HFE*-associated haemochromatosis, first symptoms occur after 30–40 years of age. Patients with the common form of hereditary hemochromatosis (HH-1, OMIM 613609) bear in more than 95% of the cases a homozygous mutation in the *HFE* gene [1] (p.(Cys282Tyr) or C282Y; rs1800562). The prevalence of the homozygous C282Y mutation that can cause hemochromatosis varies among ethnic groups but can reach 0.5% in North America and 1% in Ireland or in the French Brittany region (average heterozygosity in Europe 9.2%) [2].

A second variant, p.(His63Asp) or H63D (rs1799945) is probably not clinically relevant, but the test is still largely offered. C282Y and H63D testing is generally accepted as a first line evaluation of iron overload cause in Western Europe. Close to H63 residue is another variant, p.(Ser65Cys) or S65C (rs1800730), which is an SNP without any clinical consequence and should not be tested [3] but interferes with some H63D detection methods. Among the commercially available kits, ViennaLab provides a real-time PCR kit based on a TaqMan assay. However, the H63D probes overly the SNP rs1800730 coding the S65C polymorphism, and when present, poor hybridization led at least one (and possibly up to three) laboratory in the European Molecular Genetics Quality Network (EMQN) 2019 survey to misclassify a heterozygous H63D variant (falsely interpreted as homozygous because of an allelic dropout caused by a S65C heterozygosity). This led us to reconsider the method and develop an improved RFLP-based detection method.

We report an improvement of the PCR restriction fragment length polymorphism (RFLP) method. The method presented here is multiplexed, allowing coamplification of the *HFE* exons 2 and 4 (bearing the 63 and 282 residue codons, respectively). Codigestion is made possible by use of SexA1 for C282Y and BspHI for H63D detection. Moreover, we added amplification of a *FZD1* gene fragment carrying obligate SexA1 and BspHI sites for digestion control and two Short Tandem Repeats (SE33 and FGA) for identity monitoring and contamination tracking. Fluorescent primers allow capillary electrophoresis and accurate allele tagging.

## 2. Material and Methods

Sixty consecutive patients referred for index case analysis or familial studies were analyzed by three methods: (i) the commercial Viennalab Realtime PCR kit based on a TaqMan assay, (ii) the improved RFLP method described here, and (iii) Sanger's dideoxy sequencing as a gold standard for accurate genotyping. All patients gave informed written consent.

The QuickGene Blood DNA extraction kit was from Qiagen (Hilden, Germany). Oligonucleotides were from Eurogentec (Seraing, Belgium). SexAI and BspHI were from New England Biolabs (Evry, France). *HFE* C282Y RealFast Assay and *HFE* H63D RealFast Assay were from ViennaLab Diagnostics (Vienna, Austria). The multiplex PCR plus kit was from Qiagen (Hilden, Germany). The MasterMix PCR AmpliTaq Gold360 was from Thermo Fisher Scientific (Waltham, MA). FastAP thermosensitive Alkaline Phosphatase was from Thermo Scientific (Vilnius, Lithuania). BigDye Terminator v1.1 cycle sequencing kit and formamide were from Applied Biosystems (Austin, TX).

### 2.1. Design of the PCR RFLP-Based Method

In the original method [1], C282Y and H63D detection was based on the creation of RsaI and MboI (or Bcl I) sites, respectively. These two enzymes recognize short sequences that are very frequent in the genome. They are unsuitable for codigestion of the fragment combination described below. They were replaced by SexAI (A/CCWGGT) and BspHI (T/CATGA), respectively. The rs1800730 SNP on codon 65 (minor allele frequency 0.01) do not interfere with BspHI cleavage.

SexAI and BspHI utilization allows coamplifying exon 2 and exon 4 of *HFE* and codigestion of the PCR fragments. Codigestion was optimized by choosing a manufacturer carrying both enzymes and a universal digestion buffer. Primer pairs were designed with the Primer3 software (http://biotools.umassmed.edu/bioapps/primer3_www.cgi) and carefully chosen in the proposed sets, based on the absence (or very low frequency) of SNPs in hybridization sequences at the 3′ end of primers.

Because the putative restriction sites are unique, undigested fragments might result from accidentally undigested fragment rather than from the absence of restriction sites. Thus, an internal control was added by the mean of coamplification of an *FZD1* gene fragment encompassing one SexAI and one BspHI restriction site. Both primers were labeled allowing using this sole fragment for control of both enzymes.

The FGA STR (UniSTS240635, GenBank accession M64982), a complex tetranucleotide repeat, was amplified with published primers (https://strbase.nist.gov//str_FGA.htm accessed 03 03 2020). The SE33 STR (GenBank accession V00481) is an AAAG repeat which was amplified with primers described in https://strbase.nist.gov//str_SE33.htm. Allele calling was performed with the GeneMapper® Software version 5.0 (Applied Biosystems).

For comparison methods, 60 consecutive DNAs referred to our laboratory were analyzed by dideoxy-sequencing. Primers for amplification and Sanger sequencing were 5′ACA TGG TTA AGG CCT GTT GC and 5′GCC ACA TCT GGC TTG AAA TT for *HFE* exon 2 and 5′TGG CAA GGG TAA ACA GAT CC and 5′CTC AGG CAC TCC TCT CAA CC for exon 4. Amplifications were performed with AmpliTaq Gold 360 mastermix (Applied Biosystems), initial denaturation steps for 10 min at 95°C, then 30 cycles of denaturation at 95°C for 30 secs, hybridization at 54°C for 30 secs, and elongation at 72°C for 1 min followed by a final elongation step at 72°C for 7 min. Sequencing was performed with the FastAP thermosensitive Alkaline Phosphatase and BigDye Terminator reagents (v.1.1 cycle sequencing RR-100) according to manufacturer protocols. Dideoxy sequencing products were cleaned by gel filtration (Sephadex G25, GE Healthcare Life sciences). Sequencing reaction products were loaded onto a capillary electrophoresis apparatus (Applied Biosystems 3500 xL Dx; POP7 polymer, injection 15 secs at 1.6 kV, run 1400 secs at 19.5 kV in 50 cm capillaries).

## 3. Results

### 3.1. Initial Setup and Validation

We took advantage of the QIAGEN Multiplex PCR Kit designed for multiplex amplifications. Amplifications were performed in 10 *μ*l final volume. Each primer pair was tested in individual reactions on control DNAs (data not shown) before being mixed in multiplex reactions. After testing the initial mix at the recommended primer concentration in setup reactions (0.2 *μ*M final for each primer), we concluded it was not necessary to adjust individual primer pair concentrations to limit unbalanced amplification. Codigestions were performed with SexAI and BspHI (0.75 and 1.5 UI/*μ*l final, respectively) overnight at 37°C in the universal buffer provided by the manufacturer. The chosen final conditions are presented in Table 1. Since the primers were chosen to generate fragments markedly differing in size, many fluorochrome combinations are possible. The one reported here uses a combination of ATTO 565, Yakima Yellow, FAM, and ATTO 550 (respectively, red, green, blue, and black with the G5 filter) and is equivalent to a PET, VIC FAM, and NED combination. One microliter PCR product was added to 9 *μ*l Hi-Di formamide (Applied Biosystems) and 0.5 *μ*l size standard (GS™-LIZ® 500, Applied Biosystems) and loaded onto a capillary electrophoresis apparatus (Applied Biosystems 3500 xL Dx). Injection parameters were 1.6 kV for 7 sec, and separation was run at 19.5 kV for 1330 sec (POP7 in 50 cm capillaries).

Initial tests with AmpliTaq Gold 360 did not give satisfactory result (imbalanced amplification and incomplete non-template–directed addition of a single nucleotide to the 3′ end of a blunt-end double-stranded DNA (“plus-A-artefact”); not shown).

### 3.2. Signal/Noise

An inherent fluorescent background is present in all capillary electrophoresis runs. Fluorescence noise was measured as the highest peak in the background (blank assays with H2O loaded in formamide). Under our experimental conditions the noise was below 50 RFU. A cut-off value of 250 RFU (5 times the noise) was introduced to simplify interpretation and identification of true alleles in the optimized assay.

### 3.3. Sensitivity

DNA concentration was determined photometrically. DNAs from 4 individuals were diluted stepwise in sterile water, to concentrations corresponding to 2, 10, 20, 50, 100 ng, and 200 ng in the 10 *μ*l PCR. Under these conditions, with 2 ng of input DNA, *FZD1* digested fragments, although visible, were below the 250 RFU arbitrary threshold. At any other concentration, all peaks were in the 250-32000 RFU range, 32000 RFU being the saturation limit. When DNAs were in the 15-50 ng range per 10 *μ*l reaction, which is what is usually achieved with 2 *μ*l of DNA extracted by mean of quick extraction protocols such as the QuickGene blood test (expected value in the 25 ng/*μ*l range according to the manufacturer), satisfactory signal height and peak balance were obtained for 26 cycle amplifications (initial denaturation at 95°C for 5 min followed by 26 cycles of annealing at 60°C for 90 sec, extension at 72°C for 30 sec, denaturation at 95°C for 30 sec with a final round at 68°C for 10 min). Thus, after initial setup experiments, DNA concentration was no longer measured, and DNA input was set to 2 *μ*l, regardless of the actual concentration. One representative electrophoresis is presented in Figure 1. However, DNA assay is still mandatory when dealing with high quality DNA that will require dilution prior to amplification.

### 3.4. Specificity

Genotypes as determined by Sanger sequencing were as follows: C282Y -/-, H63D -/-, S65C -/-: *n* = 18; C282Y -/-, H63D +/-, S65C -/-: *n* = 11; C282Y +/-, H63D -/-, S65C -/-: *n* = 9; C282Y +/-, H63D +/-, S65C -/-: *n* = 8; C282Y +/+, H63D -/-, S65C -/-: *n* = 6; C282Y -/-, H63D +/+, S65C -/-: *n* = 5; C282Y -/-, H63D -/-, S65C +/-: *n* = 2; and C282Y -/-, H63D +/-, S65C +/-: *n* = 1 (+/+ and +/- refer to the homozygous and heterozygous status for the minor allele, respectively).

No discrepancy was observed on samples analyzed by dideoxy sequencing and the improved RFLP method described here (S65C status is not assessed by this RFLP method). In contrast, one sample proved by Sanger analysis to bear both heterozygous H63D and S65C variants had apparent homozygous H63D genotype when analyzed by the Viennalab TaqMan assay (apparent genotype heterozygous H63D by RFLP). The mechanism of the discrepancy is believed to be the consequence of poor hybridization of the TaqMan probe on the S65C coding allele (the variant responsible for S65C does not interfere with BspHI digestion). In this series, two other S65C variant samples were identified by dideoxy sequencing. However, although likely relying on allelic dropout, the apparent genotypes (absence of the H63D polymorphism) according to the Vienna Lab kit were correct.

### 3.5. Stutter Peaks

Amplification of STR generated artifact stutter peaks, at size equivalent to alleles but one repeat shorter than the actual allelic types. Stutter height depends on the considered STR. Stutter heights measured on a series of 40 alleles were on average 8.0% ± 2.4% and 10.6%% ± 2.4% of the allele height for FGA and SE33, respectively (m ± SD). Thus, on ongoing assays, any stutter peak above the mean + 2SD values will be regarded as resulting from contamination.

### 3.6. Contamination Detection

Coamplification of STR allows detection of contamination, whatever the mechanism involved, whereas traditional methods would only detect reagent contaminations through presence of signal in the blank control reaction.

To assess the potential for contamination detection, two DNA samples were mixed (1 : 1, 1 : 10, 1 : 25, and 1 : 100) and analyzed. Amplifications were performed with 25 ng of DNA mix. The DNA sample used for experimental contamination was deliberately chosen to have an allele with the size of the stutter of the other DNA sample. Equimolar mix gave balanced STR amplification and artificial C282Y -/- H63D +/- genotype (data not shown). Mixed DNAs at 1 : 10 ratio allowed identifying contamination either by additional STR alleles, a stutter size above the expected value and an extra H63D peak (Figure 2). Contamination and interferences were not detected in 1 : 25 and 1 : 100 dilutions.

### 3.7. Reproducibility

Reproducibility assays proved the method to be reliable. Between assays, controls (homozygous C282Y, homozygous H63D, and compound heterozygote DNAs) were systematically added, and no discrepancy has been found. Intra-assay (one sample run 10 times in the same assay) and interoperator (same control as above run at least 3 times by 4 different operators) variabilities were also checked.

## 4. Discussion

The four most frequently reported methodological approaches for C282Y and H63D typing rely on real-time PCR, PCR and restriction endonuclease digestion assay, PCR and reverse hybridization, and sequencing [4]. The S65C polymorphism is present at 1% in the general population and may interfere with H63D detection in TaqMan assays. This variant was shown here to be responsible for dropout and mistyping of a DNA sample with the Vienna Lab kit.

The initial methods for C282Y testing rely on restriction endonuclease digestion assay [1, 5]. The C282Y and H63D mutations create RsaI and MboI cleavage sites, respectively, which can be used on PCR fragments for discriminating between normal, heterozygous, and homozygous patients. This method was initially reported by Feder et al. in 1996 [1] and improved by using a new primer set [5] because of a frequent (10%) SNP in the hybridizing sequence of the original primers that leads to allelic dropout.

The primers chosen here for the RFLP method hybridize to sequences without SNPs or in the 0.0005 frequency range (dbSNP 2.0 Build 153 v2 in https://www.ncbi.nlm.nih.gov/gene/3077 accessed on May 20th, 2020). The risk of allelic dropout is limited to mishybridization in the very last 3 to 4 bases at the 3′ end of the primer. Thus, we estimate the residual risk to 1 per 100 000 compared to 1% with the Vienna Lab kit or any method relying on TaqMan probe hybridizing on the minor allele of rs1800730 SNP (S65C polymorphism).

A very elegant method was reported [6] that simultaneously detects the C282Y and H63D mutations by PCR-mediated site-directed mutagenesis and digestion using a single enzyme. The primers create a BbrPI restriction site in the wild-type sequences. However, this method also fails to correctly genotype compound heterozygous H63D/S65C individuals [7, 8], presumably because a third mismatch hampers amplification of the S65C allele.

Many enzymes are available that can differentially digest the sequences of interest. RsaI use was not possible because it digests GTCA sequences which are very frequent and spread on the amplified sequences reported here. We used SexAI instead (A/CCWGGT) and replaced MboI (formerly in use in our laboratory for H63D typing) for BspHI (T/CATGA). These enzymes are used with the same buffer and do not cut FGA and SE33 STRs. However, no internal digestion control was present. Although enzymes are mixed prior to be added in the PCR product, failure of digestion and/or enzyme distribution in the tube might occur. To overcome these difficulties, we added in the multiplex amplification an *FZD1* fragment that harbors both BspHI and SexAI sites. The identification of a sequence with these two restriction sites was facilitated by interrogation of the intronless gene database [9] http://www.bioinfo-cbs.org/igd. Fluorescent labeling of both *FZD1* primers allows using this unique fragment for both digestion controls.

Tandemly repeated DNA sequences are widespread throughout the human genome and show sufficient variability among individuals to be used in identity testing. FGA and SE33 STRs were chosen because of a high percentage of heterozygosity and because of a large allele number. For FGA, there are over 28 known alleles ranging from 12.2 to 51.2 repeats, and for SE33, there are over 76 known alleles ranging from 7 to 39.2 repeats.

The match probability for the combination of the most frequent genotypes is in the 0.0005 range with these two STRs. Inclusion of such STRs in the multiplex mix allows quality control and identity verifications. Match of the FGA and SE33 genotypes on the questioned sample and on the spared sample will demonstrate with quasi certainty that the 2 samples originate from the same individual. Moreover, in laboratories were automation has not been achieved for this analysis, duplicate distribution of a given sample instead of two different samples would be detected.

One of the major advantages of capillary electrophoresis is its precision in distinguishing fragment sizes differing by as few as a single base pair. While small differences between fragments <10 and 20 bp may be distinguished by the naked eye on agarose or polyacrylamide gels, the exact fragment size is impossible to call. Moreover, contamination, which detection is an important improvement of the present method, is at risk of being undetected if gel electrophoresis is used instead. Amplification of STR generates artifact peaks in strict repetitive patterns and stutter peaks, at size equivalent to alleles, one repeat shorter than the respective allelic types. These artifacts are believed to result from polymerase slippage during template amplification [10]. The DNA mixes used here show that once the stutter artefact has been taken care of, detection of contamination was achieved in mixes with ratio as low as 1 : 10. Moreover, interindividual contamination would be detected, whereas usual controls are generally based only on reagent contamination detection by amplification of a no DNA sample.

Although methods must always be adjusted to individual laboratories, the process reported here may be useful for other laboratories who wish to adapt this assay. In essence, the modifications involved detection in one single PCR of C282 and H63D genotypes in multiplex amplification with modified primers, thanks to the use of restriction enzymes recognizing longer sequences. The method reduces the risk of mistyping (either by contamination or interference with other SNPs). Addition of internal control for digestion and coamplification of STR allows detecting contaminations and possible sample mix ups. These advantages overcome the inconvenient of the method being a 3 steps assay (amplification digestion and electrophoresis) compared to one step TaqMan-based assays.

## Figures and Tables

**Figure 1:** Example of a compound heterozygote sample. Electrophoregram of a compound heterozygous sample (C282Y +/+, H63D +/-). (a–d) FAM-labeled PCR products (FGA STR allele), Yakima Yellow-labeled PCR products (SE33 STR alleles), and ATTO 550-labeled PCR products: FZD1 double digestion products of the FZD1 labeled on both primer size are 114 and 147 bp for SexA1 and BspHI digestion, respectively. Uncut FZD1 fragment would be 309 pb (171 or 204 bp in case of digestion failure with SexAI an BspH1, respectively). (c) ATTO 565-labeled HFE fragments digested with SexAI and BSPHI, respectively. Fragments are as labeled on the figure (H63 wild-type allele, C282Y variant, H63D variant, and C282 wild-type allele).

**Figure 2:** Contamination tracking. Two different DNAs, one C282Y -/- and H63D +/- and one C282Y -/- and H63D -/-, were mixed at a 1 : 10 ratio. In (a), an extra FGA allele is present (long arrow) corresponding to one of the FGA alleles of the contaminating DNA. Moreover, an allele the size of the stutter (in base pair) is superimposed on the stutter peak. It is detected because the size (in RFU) is above the expected stutter size. (b) The arrow points to an extra SE33 allele from the contaminating DNA. (d) The arrow points to the contaminating H63D allele.

**Table 1:** Primer sequences.

PCR primers	5′ label	Sequence (5′- > 3′)
HFE exon 2 (H63D) upper	ATTO 565	ACATGGTTAAGGCCTGTTGC
HFE exon 2 lower	—	GCCACATCTGGCTTGAAATT
HFE exon 4 (C282Y) upper	ATTO 565	CGGGCCTTGAACTACTACCC
HFE exon 4 lower	—	ACCTCCTCAGGCACTCCTCT
STR SE33 upper	Yakima Yellow	AATCTGGGCGACAAGAGTGA
STR SE33 lower	—	ACATCTCCCCTACCGCTATA
STR FGA upper	FAM	GGCTGCAGGGCATAACATTA
STR FGA lower	—	ATTCTATGACTTTGCGCTTCAGGA
FZD1 upper	ATTO 550	CTTGTCCGGCTGTTACACG
FZD1 lower	ATTO 550	CAGGATGGTGATGGTCTTGAT

PCR conditions and digestion were as follows: Qiagen multiplex PCR kit, 10 *μ*l final reaction with 15-50 ng DNA per tube; primers 0.2 *μ*M final each; initial denaturation at 95°C for 5 min followed by 26 cycles of annealing at 60°C for 90 sec, extension at 72°C for 30 sec, denaturation at 95°C for 30 sec with a final round at 68°C for 10 min; and digestion overnight with SexAI and BspHI (0.75 and 1.5 UI/*μ*l final, respectively).

## Data Availability

We state that the entire data is totally available in the article.
